The article "Monitoring of Neuroendocrine Changes in Acute Stage of Severe Craniocerebral Injury by Transcranial Doppler Ultrasound Image Features Based on Artificial Intelligence Algorithm" was retracted in 2023. Reasons: signs of a paper mill; suspected computer-generated content; unreliable results or conclusions; concerns about the data.

# Monitoring of Neuroendocrine Changes in Acute Stage of Severe Craniocerebral Injury by Transcranial Doppler Ultrasound Image Features Based on Artificial Intelligence Algorithm

**DOI:** 10.1155/2021/3584034

**Published:** 2021-12-15

**Authors:** Tao Wang, Yizhu Chen, Hangxiang Du, Yongan Liu, Lidi Zhang, Mei Meng

**Affiliations:** Department of Critical Care Medicine, Ruijin Hospital, Shanghai Jiaotong University School of Medicine, Shanghai 201801, China

## Abstract

This study was aimed at exploring the application value of transcranial Doppler (TCD) based on artificial intelligence algorithm in monitoring the neuroendocrine changes in patients with severe head injury in the acute phase; 80 patients with severe brain injury were included in this study as the study subjects, and they were randomly divided into the control group (conventional TCD) and the experimental group (algorithm-optimized TCD), 40 patients in each group. An artificial intelligence neighborhood segmentation algorithm for TCD images was designed to comprehensively evaluate the application value of this algorithm by measuring the TCD image area segmentation error and running time of this algorithm. In addition, the Glasgow coma scale (GCS) and each neuroendocrine hormone level were used to assess the neuroendocrine status of the patients. The results showed that the running time of the artificial intelligence neighborhood segmentation algorithm for TCD was 3.14 ± 1.02 s, which was significantly shorter than 32.23 ± 9.56 s of traditional convolutional neural network (CNN) algorithms (*P* < 0.05). The false rejection rate (FRR) of TCD image area segmentation of this algorithm was significantly reduced, and the false acceptance rate (FAR) and true acceptance rate (TAR) were significantly increased (*P* < 0.05). The consistent rate of the GCS score and Doppler ultrasound imaging diagnosis results in the experimental group was 93.8%, which was significantly higher than the 80.3% in the control group (*P* < 0.05). The consistency rate of Doppler ultrasound imaging diagnosis results of patients in the experimental group with abnormal levels of follicle stimulating hormone (FSH), prolactin (PRL), growth hormone (GH), adrenocorticotropic hormone (ACTH), and thyroid stimulating hormone (TSH) was significantly higher than that of the control group (*P* < 0.05). In summary, the artificial intelligence neighborhood segmentation algorithm can significantly shorten the processing time of the TCD image and reduce the segmentation error of the image area, which significantly improves the monitoring level of TCD for patients with severe craniocerebral injury and has good clinical application value.

The article "Monitoring of Neuroendocrine Changes in Acute Stage of Severe Craniocerebral Injury by Transcranial Doppler Ultrasound Image Features Based on Artificial Intelligence Algorithm" was retracted in 2023. Reasons: signs of a paper mill; suspected computer-generated content; unreliable results or conclusions; concerns about the data.

## 1. Introduction

Brain injury is defined as damage to brain tissue caused by violence acting on the head [1]. Brain injury can be divided into mild and severe brain injuries according to the degree of illness. Milder brain injury can be cured without sequelae, while the treatment of severe head injury (such as brain injury causing intracranial hematoma) can relieve symptoms and relieve life-threatening, but there are often sequelae such as amnesia, tinnitus, and vertigo [2].

Recent studies showed that many neurological complications in patients with acute severe brain injury are closely related to neuroendocrine changes, and timely and effective monitoring of neuroendocrine changes in patients is helpful to prevent neurocognitive and neurobehavioral sequelae of severe brain injury [3]. Some studies suggest that subtle neuronal injury (diffuse axonal injury) in these patients with severe brain injury can only be observed by using advanced neuroimaging, while neuroendocrine hormone levels are often used as one of the auxiliary indicators to assess the neurological injury of severe brain injury in clinical practice [4]. It was found that traumatic brain injury may cause an acute increase in stress hormones or anterior pituitary hormone deficiency, and may present with early temporary neuroendocrine abnormalities or additional late neuroendocrine abnormalities during rehabilitation [5]. In addition, the Glasgow coma scale (GCS), developed by Graham Teasdale and Bryan J. Jennett of the University of Glasgow in the United Kingdom in 1974 to determine the presence or absence of coma and the severity of coma in patients, is also widely used in clinical assessment of traumatic brain injury (TBI) severity and prediction of injury outcomes [6].

At present, the imaging examinations for brain injury in clinical practice include X-ray, CT, MRI, and ultrasonography. Among them, ultrasonography is relatively difficult for the examination of intracranial conditions due to the influence of the skull bone, while the advent of transcranial Doppler (TCD) ultrasonography largely alleviated this problem [7]. TCD ultrasonography is a means of intracranial blood flow detection using the Doppler effect. With the help of the pulsed Doppler technique and 2 MHz emission frequency, the ultrasonic beam can penetrate the thinner part of the skull and directly trace the Doppler signal of cerebral artery blood flow, so as to obtain the hemodynamic parameters of cerebral artery and reflect the cerebrovascular function status. It has the advantages of noninvasive, convenient, repeatable, and continuous and dynamic monitoring [4, 8, 9]. However, as with other ultrasound examinations, the accuracy of the acquired parameters is highly dependent on the skill of the operator and often requires a long period of training. Clinically, it is more difficult to evaluate the cerebral blood flow status of patients with acute severe brain injury, and TCD provides a good solution [10]. However, there are still some problems in the imaging clarity of intracranial conditions of TCD ultrasonography images. If the color flow signals of TCD ultrasound need to be captured by the doctor with the naked eye, it is difficult to ensure the accuracy, it is difficult to quantitatively describe the color flow signals, and it cannot visually reflect the important information related to diagnosis [11], which makes the current color Doppler ultrasound diagnosis not fully used in the diagnosis and treatment of patients with severe brain injury.

The article "Monitoring of Neuroendocrine Changes in Acute Stage of Severe Craniocerebral Injury by Transcranial Doppler Ultrasound Image Features Based on Artificial Intelligence Algorithm" was retracted in 2023. Reasons: signs of a paper mill; suspected computer-generated content; unreliable results or conclusions; concerns about the data.

In recent years, various artificial intelligence algorithms have been fully applied in the field of medical image processing [12]. For example, in the study by Lian et al. [13], an automatic segmentation method based on parameter adaptive pulse coupled neural networks (PCNN) was used for the preprocessing and preliminary segmentation of medical images such as ultrasound images of the gallbladder and gallstones and MRI images of the left ventricle, and the results showed that this algorithm had good performance. The unsupervised learning PCNN model was used for medical image segmentation of periodontal structures in a study by Wang et al. [14], which similarly achieved good results. However, there are still few reports on artificial intelligence algorithm in the field of intracranial Doppler ultrasound image processing. This study hopes to design an artificial intelligence rapid segmentation algorithm based on the characteristic information of intracranial Doppler ultrasound images of patients with severe brain injury, realizing the rapid segmentation of color vascular regions in the image and the accurate localization and extraction of the characteristic information of the injury location. In summary, this study comprehensively evaluates the application value of this algorithm by using intracranial Doppler ultrasound based on artificial intelligence rapid segmentation algorithm to monitor neuroendocrine changes in the acute phase of severe brain injury. This study provides some reference value for the study of neuroendocrine changes in the acute phase of severe brain injury while optimizing the diagnostic efficiency of intracranial Doppler ultrasonography in severe brain injury.

## 2. Materials and Methods

### 2.1. Research Objects and Grouping

A total of 80 patients with severe brain injury who were treated in the hospital from June 2018 to June 2019 were selected as the subjects, including 48 males and 32 females, aged 19-57 years. The average age was 39.32 ± 6.41 years. Among the 80 patients with severe brain injury, 41 were caused by traffic accidents, 22 by construction sites, and 17 by falls. In addition, according to the type and location of brain injury, 23 cases of acute subdural edema combined with brain contusion, 21 cases of acute epidural edema, 17 cases of multiple intracranial edema, and 19 cases of intracerebral hematoma combined with brain contusion were classified. In this study, 80 patients with severe brain injury were randomly divided into two groups. One group used conventional transcranial Doppler ultrasound images for disease monitoring, recorded as the control group, and the other group used transcranial Doppler ultrasound images based on the artificial intelligence algorithm for disease monitoring, recorded as the experimental group, with 40 cases in each group. The manufacturer of the transcranial color Doppler ultrasound equipment used in this study was Xuzhou Lianchuang Medical Equipment Co., Ltd., and the model was TCD-I (cart type). All patients were diagnosed by brain CT examination after admission and underwent acute surgery.

The article "Monitoring of Neuroendocrine Changes in Acute Stage of Severe Craniocerebral Injury by Transcranial Doppler Ultrasound Image Features Based on Artificial Intelligence Algorithm" was retracted in 2023. Reasons: signs of a paper mill; suspected computer-generated content; unreliable results or conclusions; concerns about the data.

Inclusion criteria were as follows: (1) patients who meet the clinical diagnostic criteria of severe head injury; (2) GCS score ≤ 8 points; and (3) brain injury patients diagnosed by CT (only received clinical surgery and conventional drug treatment, no hormone drug treatment). Exclusion criteria were as follows: (1) patients with severe injury of other organs; (2) patients who had liver, kidney, adrenal, thyroid, and pituitary diseases; (3) patients had endocrine and metabolic system diseases; (4) patients using hormone therapy during treatment; and (5) patients during pregnancy or lactation.

### 2.2. Neighborhood Segmentation Algorithm Model Based on Artificial Intelligence

Based on the traditional artificial intelligence convolutional neural network (CNN) algorithm, the blood flow velocity, vascular location, distribution characteristics, blood flow properties, and other information in transcranial color Doppler ultrasound images are the key indicators to monitor the intracranial conditions of patients with severe brain injury. If the color ultrasound video image is decomposed into image sequences by image analysis technology, then the valuable data relationship hidden in it is extracted. The establishment of a multiparameter and multifactor comprehensive analysis model of color ultrasound technology will significantly improve the accuracy of the diagnosis of neuroendocrine changes in patients with severe brain injury in the acute stage. Based on this, this study will use the artificial intelligence neighborhood segmentation algorithm based on the combination of domain and color clustering to segment the TCD ultrasound images of patients with severe brain injury [15].

The article "Monitoring of Neuroendocrine Changes in Acute Stage of Severe Craniocerebral Injury by Transcranial Doppler Ultrasound Image Features Based on Artificial Intelligence Algorithm" was retracted in 2023. Reasons: signs of a paper mill; suspected computer-generated content; unreliable results or conclusions; concerns about the data.

At the beginning of algorithm construction, it is necessary to realize the intelligent conversion between red, green, and blue (RGB) color space and hue-saturation-intensity (lightness) (HSI/HSL) color space on image acquisition and imaging equipment, so as to overcome the defects of color invisibility and unevenness in RGB color space [16]. Specific conversion equations are expressed as follows.

(1) $$\begin{array}{c} H=\begin{array}{cc} \cos^{-1}\left\{\frac{\left(R-G\right)+\left(R-B\right)}{2\sqrt{{\left(R-G\right)}^{2}+\left(R-B\right)\left(G-B\right)}}\right\} & B\leq G,\\ 2\pi -\cos^{-1}\left\{\frac{\left(R-G\right)+\left(R-B\right)}{2\sqrt{{\left(R-G\right)}^{2}+\left(R-B\right)\left(G-B\right)}}\right\} & B>G, \end{array} \end{array}$$

(2) $$\begin{array}{c} S=1-\left(\frac{3}{R+G+B}\right)\min\left(R,G,B\right), \end{array}$$

(3) $$\begin{array}{c} I=\frac{R+G+B}{3}. \end{array}$$

*R*, *G*, and *B* represent red, green, and blue, respectively; *H*, *S*, and *I* represent hue, saturation, and brightness, respectively. In order to measure the color difference between two points of point *a* (*H*1, *S*1, *I*1) and point *b* (*H*2, *S*2, *I*2), the Euclidean distance (*D*) is used for calculation in this study [17], and the expression is shown in the following equation.

(4) $$\begin{array}{c} D\left(a,b\right)=\sqrt{{\left(H1-H2\right)}^{2}+{\left(S1-S2\right)}^{2}}. \end{array}$$

On this basis, this study introduces the *ε* field as the characteristic measurement parameter of the gray value; an *ε* value is selected according to the overall gray distance of the image, and the adaptive *ε* value is used for the selection algorithm in the pixel field to achieve the accurate division of the *ε* field [18]. The definition of the *ε* field (*Ω*_*a*_) is expressed in Equation (5), and the calculation equation of *ε* value is expressed in Equation (6).

(5) $$\begin{array}{c} \Omega_{a}=\left\{b\in N_{a}:D\left(a\left(H1,S1,I1\right),b\left(H2,S2,I2\right)\right)\leq \varepsilon \right\}, \end{array}$$

(6) $$\begin{array}{c} \varepsilon =\frac{\sum_{a\in \text{ROI}}{\left(\text{MSE}{\left(\rho \right)}_{a}\right)}^{1/2}}{\left|\text{ROI}\right|}. \end{array}$$

*N*_*a*_ represents the natural number set, ROI represents the region of interest, *ρ* represents the domain radius, MSE(*ρ*)_*a*_ represents the mean square deviation of the domain eigenvalue of pixel *a*, and the definition of MSE(*ρ*)_*a*_ is expressed in the following equation.

(7) $$\begin{array}{c} \text{MSE}{\left(\rho \right)}_{a}=\frac{1}{\left|N_{a}\right|}\underset{b\in N_{a}}{\sum }{\left(D\left(a,b\right)\right)}^{2}. \end{array}$$

Since the hue, saturation, and brightness cannot independently complete the segmentation task when the HSI color space of the region of interest in TCD ultrasound images is segmented, it is necessary to use the similarity threshold (MEAN(*S*)_*a*_) method of chromaticity and saturation to preset the ROI region [19]. The expression is as Equation (8).

(8) $$\begin{array}{c} \text{MEAN}{\left(S\right)}_{a}=\frac{1}{\left|I\right|}\underset{a\in I}{\sum }\frac{H\left(a\right)+S\left(a\right)}{1}, \end{array}$$

(9) $$\begin{array}{c} \left\{\begin{array}{cc} \left(H\left(a\right)+S\left(a\right)>\right.\text{MEAN}{\left(S\right)}_{a} & a\in \text{ROI},\\ \left(H\left(a\right)+S\left(a\right)\right.\leq \text{MEAN}{\left(S\right)}_{a} & a\notin \text{ROI}. \end{array}\right. \end{array}$$

*H*(*α*) and *S*(*α*) represent the chroma and saturation of pixel *a*, respectively; Equation (9) is the selection equation of whether the pixel belongs to ROI. Then, the domain consistency factor is used to describe the pixel domain state. When domain consistency factor (*a*) ≥ 0.5, pixel *a* is similar to most pixels *ε* in its neighborhood, and it has a similar strength value, which means that most pixels in pixel *a* and its neighborhood belong to homogeneous regions. When domain consistency factor (*a*) < 0.5, it means that pixel *a* has a similar intensity value with a few pixels in its neighborhood. In other words, in the region adjacent to the pixel, the intensity between the pixels changes greatly, indicating that the location of the pixel should be the junction of the regions or the pixel itself belongs to the noise point. Therefore, pixels satisfying domain consistency factor (*a*) ≥ 0.5 can be defined as segmented seed pixels (SEED), which is expressed in the following equation.

(10) $$\begin{array}{c} \text{SEED}=\left\{a:\text{NCF}\left(a_{D}\right)\geq 0.5,a\in \text{ROI}\right\}. \end{array}$$

On this basis, the effective clustering and regional segmentation between seed elements and nonseed elements are quickly realized by using the equivalence relationship of similarity transfer.  Figure 1 is an example of transcranial color Doppler ultrasound segmentation based on artificial intelligence neighborhood segmentation algorithm.

The article "Monitoring of Neuroendocrine Changes in Acute Stage of Severe Craniocerebral Injury by Transcranial Doppler Ultrasound Image Features Based on Artificial Intelligence Algorithm" was retracted in 2023. Reasons: signs of a paper mill; suspected computer-generated content; unreliable results or conclusions; concerns about the data.

### 2.3. Segmentation Quality Evaluation Index of Transcranial Color Doppler Ultrasound Image Based on Artificial Intelligence Neighborhood Segmentation Algorithm

In order to measure the image segmentation accuracy of the artificial intelligence neighborhood segmentation algorithm model designed for the characteristics of craniocerebral injury in patients with severe brain injury, three different error metrics are used in this study to evaluate the segmentation accuracy of the proposed algorithm model and the classical CNN algorithm model. The three different error metrics are the false rejection rate (FRR), false acceptance rate (FAR), and true acceptance rate (TAR), and their calculation equations are expressed in the following equations.

(11) $$\begin{array}{c} \text{FP}=\frac{\left|A\cup B-B\right|}{B}, \end{array}$$

(12) $$\begin{array}{c} \text{FN}=\frac{\left|A\cup B-A\right|}{B}, \end{array}$$

(13) $$\begin{array}{c} \text{TP}=\frac{\left|A\cap B\right|}{B}. \end{array}$$

*A* is the area segmented by the measured method, and *B* is the standard area completely segmented.

### 2.4. Monitoring Index and Effect Analysis of Neuroendocrine Changes in Patients with Severe Craniocerebral Injury in Acute Stage

In this study, GCS will be used to evaluate the degree of coma in patients with severe brain injury [20]. The GCS scale includes three standard scoring systems, namely, optimal eye-opening (maximum: 4 points), optimal language response (maximum: 5 points), and optimal motor response (maximum: 6 points). The current study believes that the GCS score is a good indicator for evaluating the severity of traumatic brain injury and the prognosis of subsequent mortality. In this study, the chemiluminescent microparticle immunoassay was also used to determine the basal levels of pituitary hormones such as follicle stimulating hormone (FSH), prolactin (PRL), growth hormone (GH), adrenocorticotropic hormone (ACTH), and thyroid-stimulating hormone (TSH) in the blood of patients. The instrument used was the automatic microparticle chemiluminescent immunoassay system.

Afterwards, this study will compare the GCS score and the evaluation results of each neuroendocrine hormone level in the two groups of patients with acute severe brain injury with the results of transcranial Doppler ultrasound diagnosis and comprehensively evaluate the value of the transcranial Doppler ultrasound processed based on artificial intelligence neighborhood segmentation algorithm in monitoring the neuroendocrine changes in the acute phase of patients with severe head injury according to the degree of consistency of the comparison results. The GCS scores of each group and the occurrence probability of pituitary hormone abnormalities in patients with severe brain injury were calculated and compared with TCD ultrasound.

### 2.5. Statistical Methods

The test data were processed with SPSS19.0 statistical software. The measurement data was expressed by mean ± standard deviation ($\overset{¯}{\text{x}}\pm \text{s}$). The mean comparison between groups was performed by *t*-test, and the count data was expressed by percentage (%); *χ*^2^ test was used. When *P* < 0.05, the difference was statistically significant.

The article "Monitoring of Neuroendocrine Changes in Acute Stage of Severe Craniocerebral Injury by Transcranial Doppler Ultrasound Image Features Based on Artificial Intelligence Algorithm" was retracted in 2023. Reasons: signs of a paper mill; suspected computer-generated content; unreliable results or conclusions; concerns about the data.

## 3. Results

### 3.1. Summary of Basic Information of Two Groups of Patients

Figure 2 shows the comparison of gender distribution and average age between the two groups, and Figure 3 suggests the comparison of brain injury types between the two groups. The number of male patients in the experimental group and the control group was 27 and 24, respectively, and the number of female patients was 13 and 16, respectively. The average age of the two groups was 38.93 ± 7.32 years and 40.23 ± 5.45 years, respectively. In addition, the number of patients with acute subdural edema complicated with cerebral contusion in the experimental group and the control group was 12 cases and 11 cases, respectively. The number of patients with acute epidural edema was 11 cases and 10 cases, respectively. The number of patients with multiple intracranial edema was 8 cases and 9 cases, respectively. The number of patients with intracerebral hematoma complicated with cerebral contusion was 9 cases and 10 cases, respectively. The basic information of the two groups was compared. There was no significant difference in the average age, gender distribution, and type of brain injury between the two groups (*P* > 0.05).

### 3.2. Comparison of Transcranial Color Doppler Ultrasound Findings between the Two Groups

Figure 4 is the results of transcranial color Doppler ultrasound in the two groups. In the traditional color Doppler ultrasound images of patients with craniocerebral injury drawn by doctors with naked eyes, the division of the edge of the injury area is often quite different from the actual injury situation. After the artificial intelligence neighborhood cutting algorithm is processed, the accuracy of the edge division of the injury area in the color Doppler ultrasound images of patients with craniocerebral injury is significantly improved, and the application value of color Doppler ultrasound image in monitoring patients with severe craniocerebral injury is enhanced.

### 3.3. Running Time and Color Space Parameters of Artificial Intelligence Neighborhood Segmentation Algorithm

Figure 5 indicates the comparison of the average operation time of different algorithms. The operation time of the traditional CNN algorithm is 32.23 ± 9.56 s, while that of the artificial intelligence neighborhood segmentation algorithm for TCD ultrasound is 3.14 ± 1.02 s. Compared with the traditional CNN algorithm, the image processing time is significantly shortened, and the difference is significant, with statistical significance (*P* < 0.05).

The article "Monitoring of Neuroendocrine Changes in Acute Stage of Severe Craniocerebral Injury by Transcranial Doppler Ultrasound Image Features Based on Artificial Intelligence Algorithm" was retracted in 2023. Reasons: signs of a paper mill; suspected computer-generated content; unreliable results or conclusions; concerns about the data.

Figure 6 is the color component nominal value distribution map of TCD ultrasound image segmentation in the experimental group. The graph shows that the hue (*H*), saturation (*S*), and lightness (*I*) values obtained by converting RGB color space into HSI color space by artificial intelligence neighborhood segmentation algorithm are concentrated at 0.32, 0.94, and 0.95, respectively.

### 3.4. Comparison of Segmentation Errors of Transcranial Doppler Ultrasound Images with Different Algorithms

Figure 7 is the comparison graph of the area segmentation error of TCD ultrasound images with different algorithms. The graph shows that the FRR, FAR, and TAR of the traditional CNN algorithm are 33.312%, 0.657%, and 66.688%, respectively. The FRR, FAR, and TAR of the artificial intelligence neighborhood segmentation algorithm for TCD ultrasound are 4.924%, 3.351%, and 95.183%, respectively. Compared with the traditional CNN algorithm, the FRR of the artificial intelligence neighborhood segmentation algorithm for image area segmentation is significantly reduced, FAR and TAR are significantly increased, and the difference is statistically significant (*P* < 0.05).

### 3.5. The Accuracy Analysis of Acute Neuroendocrine Change Monitoring in the Two Groups of Patients

Figure 8 shows the incidence of GCS and pituitary hormone abnormalities in the acute stage of the two groups. The results reveal that there are 27 and 24 patients in the experimental group and the control group with GCS scores in the 6~8 range and 13 and 26 patients in the 3~5 range. There is no significant difference in the distribution of GCS scores (*P* < 0.05). The incidence rate of abnormal FSH, PRL, GH, ACTH, and TSH hormone levels in the experimental group was 73.6%, 65.3%, 94.2%, 78.5%, and 76.2%, respectively; the incidence rate of abnormal hormone levels in the control group was 71.2%, 60.1%, 92.6%, 79.7%, and 74.1%, respectively; and there was no significant difference between the two groups (*P* > 0.05).

Figure 9 shows the consistency of GCS, pituitary hormone abnormalities, and Doppler ultrasound diagnosis in the two groups. The results show that the consistency rates of GCS score and Doppler ultrasound image diagnosis results in the experimental group and the control group are 93.8% and 80.3%, respectively. The consistency rate of diagnosis results in the experimental group is significantly higher than that in the control group (*P* < 0.05). The abnormal levels of pituitary hormones FSH, PRL, GH, ACTH, and TSH in the experimental group are 78.3%, 80.5%, 90.3%, 83.1%, and 85.4%, respectively, which are significantly higher than those in the control group (57.4%, 58.6%, 72.3%, 59.7%, and 60.1%, respectively) (*P* < 0.05).

The article "Monitoring of Neuroendocrine Changes in Acute Stage of Severe Craniocerebral Injury by Transcranial Doppler Ultrasound Image Features Based on Artificial Intelligence Algorithm" was retracted in 2023. Reasons: signs of a paper mill; suspected computer-generated content; unreliable results or conclusions; concerns about the data.

## 4. Discussion

Severe head injury is a disease with high mortality and disability rate, and the pathological process is very complex. In recent years, transcranial Doppler ultrasound using ultrasonic Doppler effect to achieve the detection of intracranial vascular hemodynamics can be used for the early diagnosis of cerebral arteriosclerosis, cerebrovascular collaterals, and occlusion [21]. Especially for ischemic cerebrovascular disease caused by severe intracranial artery stenosis or occlusion, cerebral vasospasm, arteriovenous malformation, aneurysm, and carotid cavernous fistula caused by subarachnoid hemorrhage, it has high diagnostic value. TCD has the advantages of noninvasive, simple operation, and good repeatability and can be used for continuous and long-term dynamic observation of patients. However, conventional transcranial Doppler ultrasound has a certain degree of error in the changes of brain structure and hemodynamics in patients, and there are also some problems in the judgment of intracranial injury [22].

In this study, an artificial intelligence neighborhood segmentation algorithm was designed for Doppler ultrasound image characteristics of patients with head injury, and it was applied to detect neuroendocrine changes in patients with severe head injury in the acute phase. The results showed that after processing by artificial intelligence neighborhood segmentation algorithm, the accuracy of edge division of injury site in color Doppler ultrasound images of patients with brain injury was significantly improved, enhancing the application value of color Doppler ultrasound images in monitoring patients with severe head injury. However, the operation time of artificial intelligence neighborhood segmentation algorithm in processing transcranial Doppler ultrasound was 3.14 ± 1.02 s, which was significantly shorter than 32.23 ± 9.56 s of the traditional CNN algorithm, with statistical significance (*P* < 0.05) indicating that compared with the traditional CNN algorithm, the image processing time of the artificial intelligence neighborhood segmentation algorithm was significantly shortened, greatly improving the work efficiency, which was consistent with the study results of Addabbo et al. [23].

Artificial intelligence neighborhood segmentation algorithm converts RGB color space into HSI color space to obtain hue (*H*), saturation (*S*), and intensity (*I*) values concentrated at 0.32, 0.94, and 0.95, respectively. Compared with the traditional CNN algorithm, the FN of image area segmentation of artificial intelligence neighborhood segmentation algorithm was significantly reduced, FP and TP were significantly increased, and the difference was statistically significant (*P* < 0.05), thus indicating that artificial intelligence neighborhood segmentation algorithm can significantly reduce the area segmentation error of transcranial Doppler ultrasound images and more accurately intelligently identify and cut the brain injury area in Doppler ultrasound images. An improved nonlinear intensity hue and saturation (INIHS) color model was also used in the pulse convolution neural network in the report by Ganasala and Kumar [24], which significantly enhanced the contrast of medical images.

The article "Monitoring of Neuroendocrine Changes in Acute Stage of Severe Craniocerebral Injury by Transcranial Doppler Ultrasound Image Features Based on Artificial Intelligence Algorithm" was retracted in 2023. Reasons: signs of a paper mill; suspected computer-generated content; unreliable results or conclusions; concerns about the data.

The results of the diagnostic consistency of GCS and pituitary hormone abnormalities with Doppler ultrasound in the two groups showed that the GCS score of the experimental group was 93.8%, which was significantly higher than that of the control group (80.3%), and the difference had statistical significance (*P* < 0.05). The consistency rates of abnormal pituitary hormones FSH, PRL, GH, ACTH, and TSH levels with the diagnostic results of Doppler ultrasound imaging in the experimental group were 78.3%, 80.5%, 90.3%, 83.1%, and 85.4%, respectively, which were significantly higher than those in the control group (57.4%, 58.6%, 72.3%, 59.7%, and 60.1%, respectively), and the differences were statistically significant (*P* < 0.05), thus indicating that the artificial intelligence neighborhood segmentation algorithm designed in this study has a good utilization value in the monitoring of neuroendocrine changes in the acute phase of severe head injury and can well detect the neuroendocrine conditions of patients with brain injury to a certain extent from the imaging.

## 5. Conclusion

In this study, an artificial intelligence neighborhood segmentation algorithm based on the characteristics of Doppler ultrasound images of patients with craniocerebral injury is designed and applied to detect the neuroendocrine changes in patients with severe craniocerebral injury in the acute stage. The results show that the area segmentation error and running time of the Doppler ultrasound image of the artificial intelligence neighborhood segmentation algorithm are significantly reduced, and the consistency with the GCS score and pituitary hormone abnormality is significantly improved. However, there are still some deficiencies. For example, the types of neuroendocrine monitoring hormones included in this study are relatively single, mainly focusing on pituitary hormones, lacking the monitoring indicators of other neuroendocrine hormones. In this study, there are relatively few monitoring indicators used in the image segmentation quality evaluation of the designed artificial intelligence neighborhood segmentation algorithm, and more algorithm evaluation indicators will be included when further algorithm optimization will be performed in the future, and then, the application value of this algorithm will be comprehensively analyzed from multiple perspectives. In conclusion, this study confirmed that the image characteristics of the TCD ultrasound based on the artificial intelligence neighborhood segmentation algorithm have good application value in monitoring the neuroendocrine changes in patients with severe brain injury in the acute stage, which is worthy of further promotion in the clinic and provides a reference basis for the imaging diagnosis, treatment, and monitoring of patients with severe brain injury.

The article "Monitoring of Neuroendocrine Changes in Acute Stage of Severe Craniocerebral Injury by Transcranial Doppler Ultrasound Image Features Based on Artificial Intelligence Algorithm" was retracted in 2023. Reasons: signs of a paper mill; suspected computer-generated content; unreliable results or conclusions; concerns about the data.

## Figures and Tables

**Figure 1:** Image of transcranial color Doppler ultrasound segmentation based on artificial intelligence neighborhood segmentation algorithm.

**Figure 2:** Comparison of gender distribution and mean age between the two groups.

**Figure 3:** Comparison of brain injury types between the two groups.

**Figure 4:** The transcranial color Doppler ultrasound results of the two groups of patients. (a) and (c) are unprocessed TCD ultrasound images of patients in the experimental group and the control group, respectively. (b) is the ROI area map of patients with severe brain injury divided by artificial intelligence neighborhood segmentation algorithm in the experimental group. (d) is the ROI area map of brain injury in patients with (c) animated by doctors.

**Figure 5:** Comparison of average running time between two algorithms. Note: ∗ indicates significant difference compared with the control group, with statistical significance, *P* < 0.05.

**Figure 6:** Distribution map of color component nominal value by TCD ultrasound image segmentation of experimental group. Note: H: hue; S: saturation; I: intensity.

**Figure 7:** Comparison of area segmentation errors in TCD ultrasound images with different algorithms. Note: ∗ indicates that the area segmentation error of TCD ultrasound image based on artificial intelligence neighborhood segmentation algorithm is significantly different from that of the control group, with statistical significance, *P* < 0.05.

**Figure 8:** GCS score and incidence of pituitary hormone abnormalities in acute stage of two groups. Note: (a) shows the acute GCS score results of two groups of patients; (b) shows the acute pituitary hormone abnormality incidence of two groups of patients.

**Figure 9:** The diagnostic consistency of GCS and pituitary hormone abnormalities with Doppler ultrasound in the two groups. Note: ∗ indicates that the diagnostic consistency of the experimental group is significantly different from that of the control group, with statistical significance, *P* < 0.05.

The article "Monitoring of Neuroendocrine Changes in Acute Stage of Severe Craniocerebral Injury by Transcranial Doppler Ultrasound Image Features Based on Artificial Intelligence Algorithm" was retracted in 2023. Reasons: signs of a paper mill; suspected computer-generated content; unreliable results or conclusions; concerns about the data.

## Data Availability

The data used to support the findings of this study are available from the corresponding author upon request.
